# Secreted Frizzled-Related Protein 4 Inhibits Glioma Stem-Like Cells by Reversing Epithelial to Mesenchymal Transition, Inducing Apoptosis and Decreasing Cancer Stem Cell Properties

**DOI:** 10.1371/journal.pone.0127517

**Published:** 2015-06-01

**Authors:** Bhuvanalakshmi G, Frank Arfuso, Michael Millward, Arun Dharmarajan, Sudha Warrier

**Affiliations:** 1 Division of Cancer Stem Cells and Cardiovascular Regeneration, Manipal Institute of Regenerative Medicine, Manipal University, Bangalore, 560 065, India; 2 Stem Cell and Cancer Biology Laboratory, School of Biomedical Sciences, Curtin Health Innovation Research Institute, Curtin University, Perth, 6845, Western Australia; 3 School of Anatomy, Physiology and Human Biology, Faculty of Science, The University of Western Australia, 35 Stirling Highway, Crawley, 6009, Western Australia; 4 School of Medicine and Pharmacology, The University of Western Australia, Crawley, 6009, Western Australia; University of Alabama at Birmingham, UNITED STATES

## Abstract

The Wnt pathway is integrally involved in regulating self-renewal, proliferation, and maintenance of cancer stem cells (CSCs). We explored the effect of the Wnt antagonist, secreted frizzled-related protein 4 (sFRP4), in modulating epithelial to mesenchymal transition (EMT) in CSCs from human glioblastoma cells lines, U87 and U373. sFRP4 chemo-sensitized CSC-enriched cells to the most commonly used anti-glioblastoma drug, temozolomide (TMZ), by the reversal of EMT. Cell movement, colony formation, and invasion *in vitro* were suppressed by sFRP4+TMZ treatment, which correlated with the switch of expression of markers from mesenchymal (Twist, Snail, N-cadherin) to epithelial (E-cadherin). sFRP4 treatment elicited activation of the Wnt-Ca_2_^+^ pathway, which antagonizes the Wnt/ß-catenin pathway. Significantly, the chemo-sensitization effect of sFRP4 was correlated with the reduction in the expression of drug resistance markers ABCG2, ABCC2, and ABCC4. The efficacy of sFRP4+TMZ treatment was demonstrated *in vivo* using nude mice, which showed minimum tumor engraftment using CSCs pretreated with sFRP4+TMZ. These studies indicate that sFRP4 treatment would help to improve response to commonly used chemotherapeutics in gliomas by modulating EMT via the Wnt/ß-catenin pathway. These findings could be exploited for designing better targeted strategies to improve chemo-response and eventually eliminate glioblastoma CSCs.

## Introduction

Glioblastoma multiforme (GBM) is a World Health Organization Grade IV tumor and is the most common and aggressive brain tumor in adults [1]. GBM represents 15 to 20% of all primary intracranial tumors and, despite multi-modal treatment options, the overall prognosis is grim with a median survival of about 14.6 months and two-year survival of 30% [2]. The primary reasons for the poor outcomes of GBM are the high rates of recurrence and resistance to chemotherapy. The main reason for repeated recurrence and varied chemotherapeutic response has been found to be the cancer stem cells (CSCs) within the glioma tumor [3]. Glioma CSCs (GSCs) were first identified by the presence of a unique cell surface protein, prominin 1 or CD133. Subsequently, many other defining markers were identified for glioma CSCs. As with CSCs from other tumors such as blood, breast, prostate, and colon, glioma CSCs also over-express multidrug resistance (MDR) markers such as the ABC transporters, which are one of the primary causes for enhanced chemo-resistance [4].

Activated self-renewal, increased chemo-resistance, and up-regulated epithelial to mesenchymal transition (EMT), which are the characteristic hallmarks of CSCs, have been associated with aberrant Wnt/β-catenin signaling [4–6]. Several proto-oncogenes promote GBM growth and increase the CSC population by activating the Wnt pathway component, TCF-4 [7]. Secreted frizzled-related proteins, DKK1 to 4, and WIF1 prevent the initiation of Wnt signaling at the cell surface by interfering with the interaction between Wnt ligands and the FZD receptor and co-receptor LRP5-6 [8].

Secreted frizzled-related protein 4 (sFRP4) is one of five members of the sFRP family, and has been implicated to have a pro-apoptotic function in many tissues [9–15]. Over-expression of sFRP4 has been associated with a decreased rate of proliferation, decreased anchorage-independent growth, and decreased invasiveness in the prostate cancer cell line, PC-3 [16]. Silencing of the sFRP genes through hypermethylation of the promoter region has been detected in cancers such as hepatocarcinoma [17,18] and GBM [19]. In our previous reports on glioma and head and neck cancer stem-like cells, sFRP4 substantially decreased the CSC population and decreased stemness genes [20,21]. sFRP4, being a physiologically secreted inhibitor, by itself has not exhibited potent apoptotic ability in the CSCs studied. However, the role of sFRP4 appeared to be chemo-sensitizing the CSCs to commonly used onco-therapeutics to which the CSCs are refractory. In a quest to address some of the plausible causative factors by which sFRP4 could act on CSCs, we studied glioma CSCs for their response to sFRP4. We demonstrate that there is an interrelationship between EMT signature properties, chemo-resistance inducing factors, and sFRP4 mediated chemo-sensitization in glioma CSCs; thus providing a mode of action of this Wnt antagonist. This combination approach of sFRP4 and drugs holds promise for CSC-directed therapy for improving survival rate and reducing glioblastoma recurrence.

## Results

### Cancer stem cell enrichment and characterization of glioma spheres

We first enriched a CD133 positive population in the U87 and U373 glioma cell lines by growing them in spheroid cultures in the absence of serum, supplemented with growth factors LIF, EGF, and B27 in non-adherent culture plates. Spheroid colonies are a typical defining feature of CSCs, which are able to proliferate, remain undifferentiated, and retain their stemness profile in serum-free cultures. After initial cell death, a few of the remaining cells grew and proliferated rapidly, forming neurosphere colonies. Following immunohistochemistry for CD133 expression, a distinct staining of the spheroid colonies was observed. Culturing of cells in a serum-enriched monolayer culture showed low level staining for CD133 (Fig 1A). Expression of CD133 mRNA was evident only in spheroid cultures, as shown by semi-quantitative RT-PCR (S1 Fig) and quantitative PCR, which showed an increase in expression of CD133 in spheroids over the monolayer culture for both cell lines (Fig 1B). Protein expression of CD133 was observed to be higher in spheroid cultures than in the monolayer culture for both cell lines studied (S2 Fig). Finally, we characterized the presence of CD133 positive cells by flow cytometry and found that 94.12% of U87 spheroids and 83.91% of U373 spheroids were positive for CD133, whereas the monolayer culture had only 63.56% for U87 and 67.6% for U373 cell lines respectively (Fig 1C).

**Fig 1:** Analysis of cancer stem cell spheroids from U87 and U373 cell lines for expression of the CSC marker CD133 by immunocytochemistry, semi-quantitative and quantitative RT-PCR, immunoblot, and flow cytometry. a) Photomicrographs of monolayer and spheroid colonies (left panel, scale bar = 50μm, n = 3) and CD133 marker staining (right panel, scale bar = 100μm) as shown by immunocytochemistry in monolayer and spheroid colonies of U87 and U373 cell lines. b) Quantitative RT-PCR of CD133 mRNA expression of U87 and U373 cell lines grown in CSC medium. Results are the mean ± SD of three independent experiments performed in triplicates (* p value <0.05, ** p value <0.01, n = 3). ML = monolayer, CSC = cancer stem cells. c) Flow cytometry analysis of CD133 in U87 and U373 cells grown in CSC medium.

### sFRP4 suppresses growth of GSCs from U87 and U373 cell lines and heightens the response of neurospheres to temozolomide

To estimate the effects of sFRP4 and TMZ, either alone or in combination, on the growth of spheroid colonies from U87 and U373 cell lines, the 3D cultures were incubated with sFRP4 (S), temozolomide (T), or S+T for 24h. Growth inhibition was estimated by MTT, BrdU, and sphere inhibition assays. Using the MTT assay, it was observed that S or T alone inhibited proliferation of U87 and U373 spheroids by 25%. However, S+T had a greater inhibitory effect of about 50% in spheroids from both cell lines (Fig 2A). A similar pattern was observed using the BrdU cell proliferation assay, wherein S+T treatment was seen to inhibit proliferation up to 40% (Fig 2B). In untreated control cultures, the results showed that the spheroids remained intact. Treatment with S alone or T alone displayed a modest reduction in sphere size in contrast to S+T in which the disintegration of the spheres was more dramatic. This was further confirmed by labeling the spheroids for the CD133 marker by immunocytochemistry, which displayed a marked reduction of CD133 staining in S+T treated samples (Fig 2C). To estimate the percentage of inhibition and dead cells, the GSCs from U87 and U373 cell lines were subjected to propidium iodide (PI) staining after various drug treatments. The percentage of healthy cells was 83% in the untreated control, decreased marginally to 79% in S treated, with a more pronounced decrease of 68% in T treated, which decreased drastically to 27% in S+T treated GSCs from U87 cells. In GSCs from U373 cells, the untreated control had 86% healthy cells, which decreased to 55% upon S treatment. In contrast to U87 cells, T treatment and S+T treatment of U373 GSCs was seen to have a similar percentage (26%) of healthy cells (Fig 3). To determine if cell death is due to apoptosis, we studied the disruption of the mitochondrial membrane, which is an indicator of apoptosis, by using JC-1 dye [22]. The percentage of apoptotic cells increased in S, T, and S+T treated U87 and U373, thereby indicating the onset of apoptosis by changes in mitochondrial membrane potential (Fig 4). In both cell lines, the highest level of apoptosis (57% for U87 GSCs and 38% for U373 GSCs) was observed in combination treated GSCs. In order to evaluate the decrease in the CD133 positive population after drug treatment, flow cytometry analysis was performed. As expected, there was a decrease in CD133 positive cells in both U87 and U373 GSCs, the decrease being from 69% in the untreated to 62% in S treated, 54% in T, treated to 47% in S+T treated U87 GSCs, and from 68% in the untreated, 64% in S treated, 62% in T treated, to 56% in S+T treated U373 GSCs (Fig 5).

**Fig 2:** Inhibition of GBM CSCs by sFRP4 and temozolomide. a) and b) Graphs represent inhibition of U87 and U373 CSCs respectively after treatment for 24h with sFRP4- 250pg/mL (S), temozolomide- 25μM (T), and sFRP4+temozolomide (S+T). Results are the mean ± SD of three independent experiments performed in triplicates (* p value <0.05, ** p value <0.01, n = 3). c) Photomicrographs of sphere forming assay and immunocytochemical staining with CD133 after treatment with control, S, T, and S+T. Nuclei were counterstained with DAPI (blue), (scale bar = 100μm).

**Fig 3:** Propidium iodide staining. Flow cytometric analysis of the cell cycle profiles of U87 and U373 CSCs after treatment with control, S, T, or S+T after staining with propidium iodide.

**Fig 4:** JC-1 assay. JC-1 mitochondrial depolarization assay after control, S, T, or S+T treatment of U87 and U373 CSCs.

**Fig 5:** Flow cytometry of CD133 expression. Flow cytometric analysis of CD133 expression analysis of untreated, S, T, and S+T treated U87 and U373 CSCs along with control staining with iso PE.

### sFRP4 down-regulates EMT promoting genes and chemo-resistance genes

Analysis by semi-quantitative and quantitative RT-PCR was used to determine the expression changes of CD133, EMT markers, and drug resistance genes. Treatment of U87 and U373 GSCs with sFRP4 and TMZ resulted in a significant increase in expression of the epithelial marker E-cadherin. The expression of the mesenchymal marker N-cadherin was observed to have reduced significantly in S+T treated GSCs, with a pronounced decrease in U87 GSCs. A decrease in the stemness related marker CD133 was observed to be dramatic in S+T treated GSCs from U87 and U373 cell lines. To assess if the structural changes of EMT were reflected in changes of the transcriptional regulators of EMT, the expression of *Snail*, *Twist*, and *Slug* was studied. Expectedly, treatment with S+T led to a significant decrease in expression of these three transcription factors in both cell lines as seen by RT-PCR (S3 Fig) and qPCR (Fig 6A and 6B). These results clearly point to changes related to EMT at the molecular level. To analyze if the drug sensitivity was accompanied by a decrease in the expression of drug transporters, expression studies were performed on *ABCG2*, *ABCC2*, and *ABCC4*. It was observed that expression of these markers reduced significantly upon treatment with S+T, and the level of *ABCC2* was undetectable in S+T treated U87 GSCs (Fig 6A and 6B).

**Fig 6:** EMT promoting and ABC transporter genes are down-regulated in CSCs treated with sFRP4 and temozolomide. a) and b) Representative graphs showing relative mRNA expression of CSC marker, EMT-related genes (*N-cadherin*, *Twist*, *Snail*, and *Slug)*, and drug transporting genes (*ABCG2*, *ABCC4*, and *ABCC2*) in U87 (a) and U373 (b) CSCs after drug treatment was performed by quantitative RT-PCR. Results are the mean ± SD of three independent experiments performed in triplicates (* p value <0.05, ** p value <0.01, n = 3).

### sFRP4 down-regulates fibroblastic markers of EMT and activates Wnt/calcium pathway

The typical changes observed during EMT include less intercellular adherence, fewer tight junctions, and loss of cellular polarity. β-catenin activation and co-expression of fibroblastic markers vimentin and α-smooth muscle actin (α-SMA) are cellular events accompanying these changes [23].

We investigated the expression of the three EMT related markers, β-catenin, α-SMA, and vimentin at the protein level. In U87 spheroid cultures treated with different drug combinations, the cells expressing α-SMA, vimentin, and β-catenin were analyzed by immunohistochemical localization. The spheroid cultures lost their spherical morphology, and the expression of α-SMA and vimentin in S+T treated cells was weak. The cells had undergone massive cell death, sphere disruption, and were adherent in S+T treated U87 spheres; and the proportion of β-catenin staining cells was very low in comparison to the untreated control spheroid cells (Fig 7A). The pattern observed by immunohistochemical staining was further confirmed by Western blotting. Treatment of U87 spheroids with S+T resulted in a substantial reduction in α-SMA, vimentin, and β-catenin protein expression when compared to the untreated control U87 spheroid cells (Fig 7B).

**Fig 7:** Treatment of CSCs with sFRP4 results in down-regulation of functional mesenchymal protein expression. a) Immunocytochemistry of mesenchymal markers α smooth muscle actin (α SMA), vimentin, and ß-catenin in U87 CSCs treated with control, S, T, or S+T (scale bar = 100μm). Nuclei were counterstained with DAPI (blue). b) Immunoblot analysis of α SMA, vimentin, and ß-catenin in U87 CSCs treated with control, S, T, or S+T.

We next investigated the effect of sFRP4 on the non-canonical arm of Wnt signaling via the mobilization of intracellular Ca_2_^+^. The effect of sFRP4 on the Wnt/calcium signaling pathway in CSCs was examined using a fluorescent indicator FURA-2. After treatment with sFRP4, there was a significant increase in intracellular Ca_2_^+^ release (Fig 8), thereby suggesting an involvement of non-canonical Wnt signaling in sFRP4 mediated inhibition of CSCs.

**Fig 8:** Fura-2 calcium assay. Intracellular calcium assay determined by fluorescent radiometric Ca_2_^+^ indicator Fura-2, in U87 CSCs treated with control, S, T, or S+T (* p value <0.05, ** p value <0.01, n = 3).

### Spheroid cells display lower colony forming ability, Extracellular Matrix (ECM) penetration, and migratory/invasive potential after treatment with sFRP4 and temozolomide

Rapid self-renewal is the hallmark property of CSCs, and the loss of stemness results in differentiation and exit from the cell cycle. As an analogy, we studied the self-renewal trait as an indicator of inhibition or apoptosis of CSCs. By sphere-forming assays in soft agar, we compared the ability to form spheres in untreated control, S, T, and S+T treated U87 spheroids. By staining the colonies with crystal violet, it was observed that untreated GSCs formed large colonies, but in S alone and T alone treated cells, the colonies were smaller and proliferation was weak. In addition, in U87 GSCs treated with S+T, the colonies had a drastic decrease in size and the cell numbers in the colonies were meager (Fig 9A).

**Fig 9:** sFRP4 and temozolomide treatment of CSCs leads to the down-regulation of invasiveness, migratory, and colony forming potential. a) Micrograph images of soft agar colony assay of U87 CSCs after treatment with control, S, T, or S+T. Staining with crystal violet indicated the colony size (scale bar = 50μm). b) Angiogenic assay of U87 CSCs (treated for 24h with control or S, T, or S+T) seeded on a pro-angiogenic ECMatrix gel pre-coated plate. Staining with crystal violet detected tube formation and initial processes (scale bar = 100μm). c) After treating U87 CSC with control, S, T, or S+T for 24 hr, an *in vitro* transwell migration assay was performed. Crystal violet staining indicated cell migration across the transwell chamber (scale bar = 100μm).

The primary ability of CSCs is the capacity to initiate the growth of the primary tumor and drive invasion and metastasis. There is an established relationship between the percentage of CSCs in breast cancer and the manifestation of metastasis [24]. The invasive ability can be correlated to the cells’ ability to penetrate and proliferate through the ECM. We examined the ability of U87 GSCs to grow on an ECM and the subsequent inhibition of this property by drug treatment. It was observed that, in the S+T treated GSCs, the proliferation was hampered after 24h of equal cell seeding (Fig 9B, panel 2). Staining with crystal violet revealed a clear inhibition of cell growth through the ECM in S+T treated cells (Fig 9B, panel 3). Invasion leads to metastatic spread and we investigated this by comparing the metastatic potential of various drug treated U87-GSCs using a Matrigel invasion chamber. We observed a dramatic difference between untreated and S+T treated cells, as the untreated cells migrated completely through the membrane and aggregated as colonies. The migratory potential of S+T treated cells was severely hampered and it was observed that only a few cells with differentiated morphology had migrated (Fig 9C).

### tumorigenic potential *in vivo* decreased after treatment of U87 GSCs with sFRP4 and temozolomide

To determine the level of tumorigenicity of U87 GSCs after treatment with S, T, and S+T, we observed tumor development in nude mice that had been injected subcutaneously with tumor cells. On the 4^th^ day of injection, animals receiving no treatment developed tumors, while animals receiving S+T treated GSCs had no tumor formation. GSCs treated with T had a smaller tumor when compared with S treated GSCs, but both were smaller than the untreated control at the 4^th^ day of injection (Fig 10A). On the 10^th^ day, upon harvest, there were significantly smaller volumes of subcutaneous tumors from the mice injected with S+T treated GSCs than that of untreated, S treated, and T treated groups (Fig 10B).

**Fig 10:** CSCs treated with sFRP4 and temozolomide possess lower tumorigenic potential *in vivo*. Average tumor size (a, b) after subcutaneous injection of U87 CSCs treated with control (U), S, T, or S+T (* p value <0.05, ** p value <0.01, n = 4).

## Discussion

Glioma stem cells can be obtained by different strategies such as cell sorting based on surface markers such as CD133, enrichment of the dye effluxing side population, and the drug and radiation resistant cell populations expressing ATP-binding cassette transporters and ATM proteins respectively [25,26]. In the present study, we enriched CSC populations from two human glioblastoma cells lines, U87 and U373, by growing spheroids in serum-free cultures and confirmed the CSC property by virtue of their pronounced elevation of CD133 expression. Using enriched glioma stem cells from these two glioma cell lines, we studied their inhibition by chemotherapeutics, augmented by sensitization with sFRP4. We could clearly demonstrate that a combined treatment of sFRP4 with the standard drug used for GBM, temozolomide, inhibited proliferation of GSCs from both cell lines, disrupted their sphere formation ability, decreased their colony formation in a soft agar assay, and impeded cell cycle progression as evidenced by PI staining. Depolarization of the mitochondrial membrane is a clear indicator of apoptosis where the integrity of the mitochondrial membrane is compromised [22]. We could clearly show a pronounced mitochondrial membrane disruption in the drug treated GSCs.

To determine the tumorigenic potential of the drug treated GSCs *in vivo*, tumor development was performed in nude mice. The results and the patterns of *in vitro* experiments were further confirmed *in vivo*, wherein S+T combination-treated GSCs had the smallest volumes of subcutaneous tumors. Chemo-sensitization is one strategy to overcome chemo-resistance and involves the use of one drug to enhance the activity of another by modulating the mechanisms of chemo-resistance. Our studies show that sFRP4 potentiated the effect of TMZ on glioma stem cells. Wnt signaling is a key pathway involved in normal tissue homeostasis. The sFRPs are the largest family of secreted Wnt antagonists and are homologous to the ligand-binding cysteine-rich domain of the Frizzled family of Wnt receptors. sFRP4 is involved in the regulation of apoptosis, proliferation, tissue formation, and tumor growth [10,12,27,28]. Chemo-sensitization by sFRP4 will serve dual purposes: decreasing the required chemotherapeutic load to the cancers and promoting a sustained Wnt inhibition in order to provide a therapeutic window for chemotherapy, while sparing the normal Wnt-dependent tissues. This dual advantage could prevent prolonged use of both Wnt antagonist and temozolomide, and sidetrack the undesirable toxic effects of therapy on normal cells.

Activation of epithelial to mesenchymal transition is essential for efficient metastatic colonization, and it is a process actively up-regulated in CSCs. The emerging, defining feature of CSCs is the acquisition of mesenchymal traits and the transition from the epithelial to the mesenchymal phenotype [29]. In this study, we present an insight into the mechanism of inhibition of CSCs by sFRP4 by analyzing the epithelial and mesenchymal properties of glioma stem cells after chemo-sensitization with sFRP4. Non-adherent sphere forming assays are reliable assays used to evaluate stem cell activity in normal tissue and putative CSCs, and the neurosphere is a well-studied sphere assay [30]. We observed that GSCs treated with S+T had substantially increased anchorage and decreased sphere forming ability, wherein the cells could grow out of the spheres and adhere to form a monolayer. In a similar study in CSCs from head and neck carcinoma, spheroid cultures where shown to over-express EMT markers and had decreased spheroid formation ability, and the increased adherence was proportional to the mesenchymal to epithelial switch [31]. Another typical phenotypic manifestation of EMT is migration and invasion [32,33]. We observed that treatment with S+T decreased GSC invasiveness through ECM and migration through transwell chambers, which could be interlinked to the acquisition of epithelial traits by this drug combination.

Increase in adherence and anchorage is accompanied by the manifestation of the epithelial marker E-cadherin, desmosomes, and the tightening of adherens junctions, which are anchored to the cytoskeleton by ß-catenin; and by the loss of mesenchymal defining markers such as the cytoskeletal proteins vimentin and smooth muscle actin [34]. This is accompanied by a transcriptional shift of factors that activate mesenchymal genes and suppress epithelial markers such as Snail, ZEB, and the bHLH family of transcription factors, and increase the deposition of the ECM protein, fibronectin. The pronounced reduction that we observed of the cytoskeletal proteins, vimentin, and α smooth muscle actin, and the adherens junction protein, ß-catenin, in S+T treated CSCs is clear testimony to the switch of the status from mesenchymal to epithelial.

The members of the Snail family- Snail, Slug, and Smuc, have a common SNAG domain and a zinc finger region at the C-terminus through which they bind to E-boxes in the promoter regions of target genes. The Snail family of transcription factors initiates the repression of E-cadherin by mediating histone modifications, which alter their protein stability and intracellular localization. Regulation of Snail proteins is under the control of various signals including Wnt, Shh, EGF, FGF, and TGFβ [35]. The transcription factor Twist interacts with components of the NuRD complex, polycomb repressor complexes PRC1 and PRC2 on the E-cadherin promoter and represses E-cadherin, whereas binding of Twist 1 to methyltransferase SET8 activates N-cadherin. The involvement of EMT-mediating transcription factors were clearly seen in our study where the expression of *Snail*, *Slug*, and *Twist* decreased to half in S+T treated GSCs. In concordance, the expression of the functional epithelial marker E-cadherin had a two fold increase in S+T treated GSCs, and its mesenchymal counterpart N-cadherin decreased upon drug treatment.

sFRP4 has a multi-level action on the Wnt/ß-catenin pathway and can antagonize the Wnt/ß-catenin and also the non-canonical Wnt/planar cell polarity pathway by activating the Wnt/Ca_2_^+^ pathway [36]. The accumulation of Ca_2_^+^ by sFRP4 that we observed in our studies could indicate activation of calcineurin, which has been shown to be stimulated by sFRP2 via the Wnt/Ca_2_^+^ pathway [37]. Calcium has been implicated to be an important mediator of antagonism of Wnt signaling by acting at multiple points. An increase in intracellular calcium results in the activation of calcium/calmodulin dependent protein kinase II (CamKII) and protein kinase C (PKC), which in turn antagonizes the canonical Wnt pathway [38,39]. The resultant apoptosis that we observed after sFRP4 treatment could thus be an effect of increased intracellular calcium levels and, in turn, the increase in calcium could increase reactive oxygen species (ROS), and ROS can induce apoptosis [36].

CSCs play an integral role in tumor recurrence by virtue of their enhanced chemo-resistant properties. Chemo-resistance is manifested at the molecular level by the expression of drug transporters, namely the ATP binding cassette (ABC) proteins associated with multiple drug resistance [40,41]. Furthermore, an association between the transcription factors regulating EMT and over-expression of drug transporters has been established [42]. Hence, the decreased expression of drug efflux proteins ABCG2 and ABCC4 by S+T treatment may reflect the gain of epithelial characteristics, and that the two processes of EMT and chemo-resistance may be intertwined.

In summary, in this study we provide evidence that the endogenously expressed Wnt antagonist, sFRP4, aids in chemo-sensitizing glioma stem cells to the commonly used glioma chemotherapeutic agent, temozolomide. Our data provide insights into the molecular mechanisms underlying this effect of sFRP4, suggesting that sFRP4 acts through altering the closely intertwined and complex CSC properties of self-renewal, epithelial to mesenchymal transition, and drug effluxing machinery, which we have summarized in a schematic representation (S4 Fig). Combination treatment of sFRP4 with conventional chemotherapeutics will help reduce the chemotherapeutic load, which is significant from a clinical standpoint. Our data suggest that targeting the Wnt pathway could inhibit the pro-survival signals of CSCs within the glioma on the one hand, and retard invasion and migration on the other, thereby preventing tumor metastasis and relapse.

## Materials and Methods

### Cell culture

Human glioblastoma cell lines U87 and U373 were obtained from the National Center for Cell Sciences, Pune, India, and maintained in DMEM/F-12 and DMEM-HG (Gibco) (1:1), containing 1X GlutaMax (Life Technologies), 10% Fetal Bovine Serum (HiMedia), and 100U/mL PenStrep (Life Technologies). Serum free medium (SFM) for sphere culture was performed in basal medium (DMEM/F-12 + DMEM-HG) with 100U/mL PenStrep, 2mM GlutaMAX, and containing 20 ng/mL each of epidermal growth factor (EGF), basic fibroblast growth factor (bFGF; R&D Systems), and leukemia inhibitory factor (LIF; Chemicon). All cells were cultured at 37°C in a humid incubator with 5% CO_2_.

### Immunofluorescent staining

For early characterization of the CSC marker, CD133, immunofluorescent (IF) staining of spheres derived from U87 and U373 cell lines cultured in CSC medium was performed. For further analysis of U87 and U373 CSCs after drug treatment, IF staining was undertaken to investigate α-SMA, vimentin, and ß-catenin expression as previously described [43]**,** with some modifications. Briefly, cells were fixed using 4% paraformaldehyde for 20 min at 4°C, and blocked with 3% bovine serum albumin (BSA) in PBS for 30 min at room temperature. The cells were then incubated for 1h in dark conditions at 4°C with primary non-labeled mouse anti-human antibodies against CD133, α-SMA, vimentin, and ß-catenin (1:200 dilutions, BD Biosciences), followed by anti-mouse rabbit fluorescein isothiocyanate (FITC) or phycoerythrin (PE) labeled secondary antibodies (1:500 dilutions, Invitrogen) for 1h at 37°C. The nucleus was counter-stained with 4’,6-diamidino-2-phenylindole (DAPI) (1:10 000 dilution) and a drop of anti-fade (Vectashield; Vector Laboratory, Burlingame CA, USA) was added to avoid quenching of the fluorochrome before placing the cover slip. The slides were visualized using a Nikon Eclipse TE2000-U fluorescent microscope and photographs were taken using Qimaging- QICAM-fast 1394.

### Western blotting

The expression of CD133 protein was confirmed by Western blotting. After drug treatment of CSCs from U87 and U373 cell lines, protein levels of epithelial and mesenchymal markers, α-SMA, vimentin, and ß-catenin were studied. Equal amounts of cell lysate proteins were separated by SDS-PAGE, transferred to polyvinylidene difluoride membranes (Millipore), and detected with CD133, α-SMA, vimentin, and ß-catenin monoclonal antibodies (mAbs) at 1:500 dilution, (R & D Systems, MN, USA) with GAPDH mAb at 1:1000 dilution (Millipore) as a housekeeping control. Rabbit anti-mouse horseradish peroxidase-linked secondary antibodies (1:3000) were used to bind to the primary antibody. The blot was developed with enhanced chemiluminescence reagent (Pierce, IL), and images were captured using AlphaImager (CA, USA).

### Flow cytometry

The percentage of CSCs expressing CD133 was determined by flow cytometry to validate the enrichment of CSCs in U87 and U373 CSC cultures. The decrease in the CD133 positive CSC population was determined after drug treatment in both U87 and U373 CSC cultures. Cell cycle perturbations after drug treatment were analyzed by propidium iodide (PI) DNA staining according to a previously reported protocol [44]. Briefly, CSCs from U87 and U373 cell lines were treated with sFRP4 (S; 250pg/ml) (R and D Systems, Australia) or temozolomide (T; 25μM) (Sigma (St Louis, MO, USA), or S+T for 48h. Then cells were centrifuged at 1000 rpm for 10 min, washed twice with PBS, and fixed in pre-chilled 70% ethanol. After fixing, the CD133 positive population was determined by incubation with mouse anti-human FITC labeled antibodies against CD133 (1:100 dilution, BD Biosciences) for 1h on ice. Cell cycle analysis was performed as previously published [45]. Briefly, after fixation, the cell pellets were suspended in 1 mL of PBS containing 0.02mg/mL of propidium iodide, 0.5mg/mL of DNase-free RNase A, and 0.1% of Triton X-100 and incubated at 37°C for 30 minutes. The cells were acquired using a BD-FACS Calibur flow cytometer with a 488nm laser, and data were analyzed by Cell Quest Software (Becton Dickinson, San Jose, CA, USA).

### Proliferation assays

#### MTT

The TACS MTT assay kit (R&D Systems) was used according to the manufacturer’s protocol to measure cell metabolic viability. Glioma lines U87 and U373 were cultured under CSC conditions (10 000 cells/mL) in 96-well plates following a published protocol [20,21]. Briefly, 10000 cells/mL were seeded in ultralow-adherent 96-well plates and incubated in CSC media for 48h. Cells were then treated with S (250pg/ml) or T (25μM) or a combination of these drugs (S+T), as well as including an untreated (U) control group for 24h. After the drug treatment, an MTT assay was performed and the plates were read at 595 nm using a Victor 3 Multilabel Plate Reader (Perkin-Elmer).

#### BrdU assay

For detecting the number of actively proliferating cells, a BrdU assay was performed in CSC enriched U87 and U373 cells, subjected to the drug treatments S, T, and S+T and compared to untreated control U. After 24h treatment, cell proliferation was measured using the BrdU Cell Proliferation Assay Kit (Cell Signalling Tech Inc) according to the manufacturer’s protocol. Plates were read at 450nm using a Victor 3 Multilabel Plate Reader.

#### JC-1 mitochondrial membrane potential assay

The rate of mitochondrial membrane disruption due to drug treatment was analyzed by using a MitoProbe JC-1 Assay kit (Invitrogen) followed by flow cytometry as described previously [46]. CSC enriched U87 and U373 cells were treated with drugs S, T, and S+T for 24hrs and compared with untreated control. After treatment, cells were harvested and washed thrice in warm PBS and subjected to 2 μm JC-1 and incubated at 37°C, 5% CO_2_ for 30min. The stained cells were washed once in warm PBS, centrifuged and resuspended in warm PBS, and analyzed on a Cell Quest Software (Becton Dickinson, San Jose, CA, USA) flow cytometer to detect fluorescence at excitation/emission wavelengths of 485/530 nm respectively.

### RNA extraction and RT-PCR

Total RNA was extracted from U87 and U373 CSCs after drug treatment using Trizol reagent (Invitrogen, USA) according to the manufacturer’s instructions. CSCs from both cell lines were first confirmed for the over-expression of CD133 by qualitative and quantitative RT-PCR. CSCs were then subjected to drug treatments U, S, T, and S+T for 24h. After treatment, cells were washed and pelleted, and total RNA and 200ng of RNA was reverse transcribed using the RevertAid First Strand cDNA Synthesis Kit (Thermo scientific) according to the manufacturer’s instructions. Briefly, total RNA was mixed with 1 μL Oligo dT (50 μM) and 1 μL of dNTP (10mM), made up to 13 μL with DEPC treated water, and heated at 65°C for 10 minutes, followed by incubation on ice. After primer hybridisation, 7 μL reaction volume containing 5X first strand buffer, RNase OUT (40U/μL), 0.1 M DTT, and Superscript III were added to the RNA and subjected to thermocycling (25°C, 5 min; 50°C, 60 min; 70°C, 15 min). PCR was carried out under the following conditions: 5min denaturation at 94°C, renaturation for 30 cycles at 94°C for 30s, 57°C for 30s, 72°C for 30s, and 7 min extension at 72°C in a Veriti 96 well thermal cycler. Qualitative expression of markers for CSCs, apoptosis, drug resistance, and EMT (primers from Sigma, sequence as indicated in the Table 1) were analyzed by PCR (95°C 30s; annealing temperature, 30s; 72°C 30s for 40 cycles) in a Veriti 96 well thermal cycler. Products were resolved using 1.5% agarose gel electrophoresis and detected using ethidium bromide. Equal loading was confirmed by the expression of the internal control gene *GAPDH*, and visualized in UV light using Alpha Imager.

**Table 1:** Primer sequences for CSC marker, EMT and drug resistance associated genes.

Genes	Primers	Base pair	Annealing temperature °C
CD133	F—5’ TCAGTGAGAAAGTGGCATCG 3’R—5’ TGTTGTGATGGGCTTGTCAT 3’	313	60
Twist	F—5’ CAGCGCACCCAGTCGCTGAA 3’R—5’ CGCCCCACGCCCTGTTTCTT 3	438	53
Snail	F—5′ GAGGCGGTGGCAGACTAG 3′R- 5′ GACACATCGGTCAGACCAG 3′	159	60
Slug	F—5’ TGCGATGCCCAGTCTAGAAA 3’R—5’ GTGTCCTTGAAGCAACCAGG 3’	160	60
N-cadherin	F—5′ CTCCTATGAGTGGAACAGGAACG 3′R—5′ TTGGATCAATGTCATAATCAAGTGCTGTA 3	121	63
E-cadherin	F—5′ ATTCTGATTCTGCTGCTCTTG 3′R—5′ AGTAGTCATAGTCCTGGTCTT 3′	400	60
ABCG2	F—5’ CACAGGTGGAGGCAAATCTT 3 ‘R—5’ CCGAAGAGCTGCTGAGAACT 3’	199	60
ABCC4	F—5’ CCATCTGTGCCATGTTTGTC 3’R—5’ AGGGCTGAGATGAGGGAACT 3’	403	59
ABCC2	F—5’ AGAGCTGGCCCTTGTACTCA 3’R—5’ TGCGTTTCAAACTTGCTCAC 3’	492	60
GAPDH	F—5’ CAGAACATCATCCCTGCATCCACT 3‘R—5’ GTTGCTGTTGAAGTCACAGGAGAC 3’	181	61

The mRNA expression of different genes obtained qualitatively was further quantified using the KAPA qPCR SYBR green PCR Master Mix (Geneworks, Australia) in a real time PCR system. cDNAs and gene-specific primers were mixed with 2X iQ SYBR Green Supermix (Bio-Rad), and dispensed on a MicroAmp Optical 8-Tube Strip. Fluorescence shift was observed using a 7500 Real-time PCR system (Applied Biosystems). Reaction parameters were 50°C for 2 minutes, 95°C for 10 minutes, followed by 40 cycles of 95°C for 15 seconds and 60°C for 1 minute. PCR products were verified by melting curves. The relative abundance of target gene mRNAs was obtained using the comparative cycle threshold method and was normalized to the internal control gene *GAPDH*, and ΔCT was calculated by subtracting the CT value of the *GAPDH* reference gene from that of each target gene. Results were also expressed as fold changes (ΔΔCT) in the mRNA levels of a target gene compared to the treated or untreated samples.

### Functional analysis of the mechanism of action *in vitro*

#### Determination of intracellular calcium

The increase in intracellular calcium levels after exposure of CSCs to sFRP4 was determined using the fluorescent radiometric Ca_2_^+^ indicator Fura-2 acetoxymethyl ester (Fura-2, 1μ mol/L, Molecular Probes) as previously reported [47]. U87 and U373 CSCs were treated with plain medium or S, T, or S+T for 24h and, after washing the cells, Fura-2 (1μ mol/L, Molecular Probes) was added to the cells in plain medium and incubated for 37°C for 45 min. Fluorescent intracellular Ca_2_^+^ flux was identified by fluorescence microscopy (450–480nm) and calorimetrically at 480nm.

#### Soft agar colony forming assay

For observing the self-renewing capacity after treating CSCs with a combination of drugs, a soft agar assay was used to determine the colony formation of tumorsphere cells under anchorage-independent conditions. CSCs from the U87 cell line were treated with plain medium, S, T, or S+T for 24h. After treatment, the neurospheres were pelleted and washed with PBS and disrupted into single-cell suspensions. Six-well plates were coated with 1 mL of 10% FBS DMEM-F12 medium with 1% agarose. After 20 min of incubation at 37°C, equal numbers of cells (1000) were plated in each well in medium with 0.5% agarose. Cells were incubated for 14 days under standard conditions (37°C, 5% CO_2_) for the formation of colonies, with the addition of 300mL of medium every 3 days to hydrate the exposed agarose. At the end of the incubation period, wells were examined under a light microscope and the colonies were further visualized by crystal violet staining (0.05%), and photographs were taken using Qimaging- QICAM-fast 1394s.

#### Extracellular matrix (ECM) angiogenesis assay

The ability of U87 CSCs to form capillary tubes after various drug treatments was investigated using an In-vitro angiogenesis assay kit (Millipore, USA) according to the manufacturer’s instructions. The formation of capillary tubes by the U87 cell line in Matrigel has been previously demonstrated [48]. CSCs from the U87 cell line were treated with plain medium, S, T, or S+T for 24h. After treatment, an equal number of cells (10 000 cells/well) were seeded on an ECMatrix gel pre-coated 96-well plate. After 24h, the cells were stained with crystal violet (0.05%) and capillary tube formation was observed by bright field phase contrast microscopy (Nikon- Eclipse TE 2000-S), and photographs were taken using Qimaging- QICAM-fast 1394. The experiments were repeated thrice.

#### *In vitro* migration assay

To study the effect of sFRP4 treatment on CSCs from the U87 cell line, cell migration was analyzed using a Transwell Migration System (BD Biosciences). After treatment of U87 CSCs with S, T, S+T, or plain medium for 24h, the neurospheres were washed, pelleted, and disrupted into single cell suspensions. Equal numbers of cells (10 000 cells) were plated into the upper chambers (Transwells with 8.0 μm pore size) in plain control medium. The lower compartment of the chamber contained 1mL of plain medium. The chambers were cultured at 37°C in 5% CO_2_ for 12 hours. The filter membranes were removed and cells that had migrated to the lower surface were fixed with 95% methanol for 5 min and stained with crystal violet (0.05%) before visualization with a phase contrast microscope (Nikon- Eclipse TE 2000-S). The experiments were performed in triplicates.

### *In vivo* tumorigenesis

U87 CSCs were sub-cutaneously implanted into nude mice as described previously [49]. All animal experiments were performed at Anthem Biosciences Ltd, Bangalore, India after approval by the Institutional Animal Ethics Committee of Anthem Biosciences and Manipal University. Briefly, U87 cells were grown under CSC conditions. The resulting neurospheres were subjected to the following treatments- U, S, T, and S+T for 48h. After the treatment duration, cells were washed thrice with PBS and centrifuged. The resulting pellet was resuspended in 1% methylcellulose in serum-free DMEM at a concentration of 1 X 10^6^ per 100 μL. Male athymic nude mice were used in this study and were housed under standard laboratory conditions, in environmentally monitored air-conditioned room with adequate fresh air supply, room temperature 22 ± 3°C and relative humidity 30–70%, with 12 hours fluorescent light and 12 hours dark cycle. Total numbers of animals used in the study were 16. Animals were observed at least once daily by the staff veterinarian to assess any adverse clinical signs during the study. Subcutaneous implantation of cells was performed in the mice under anaesthesia using isoflurane to minimize pain, and tumors were established by subcutaneous injection of 100 μL of cell suspension into the right flank. The tumors were palpable after 2 days and grew in size up to 10 days. The maximum size of tumor reached was 120 mm^3^. Tumors were excised after the 10^th^ day and examined. Animals were euthanized by CO_2_ asphyxiation prior to tumor removal.

### Statistical analysis

Data are represented as mean and SE from experiments performed in triplicate. Statistical significance was assessed by a two-sided Student’s t test. For all statistical analyses, probability values of <0.05 were considered significant (* p value < 0.05).

## Supporting Information

S1 Fig Semi-quantitative RT-PCR of CD133 mRNA expression when U87 and U373 cell lines were grown in monolayer condition or in CSC medium. (TIFF)

S2 Fig Immunoblotting of CD133 protein levels when U87 and U373 cell lines were grown in monolayer condition or in CSC medium. (TIFF)

S3 Fig RT-PCR analysis of EMT genes *E-cadherin*, *N-cadherin*, *Slug*, *Twist*, and Snail and drug transporting ABC genes *ABCG2* and *ABCC4* in untreated, S, T, or S+T treated U87 and U373 CSCs. (TIFF)

S4 Fig A schematic representation of the effect of sFRP4 on glioma stem cells. The transition from an epithelial to the mesenchymal (EMT) morphology of glioma stem cells is characterized by an up-regulation of vimentin and αSMA. Glioma stem cells have an over-expression of multidrug resistance markers and stemness markers, which are regulated by the activation of the Wnt pathway. This results in the activation of the drug efflux pumps such as ABCG2, ABCC2 and ABCC4, which increases drug resistance. sFRP4, the Wnt antagonist, inhibits this process by binding to the Fzd receptor and Wnt ligand by the canonical pathway through ß-catenin and up-regulates the non-canonical Wnt-Ca_2_^+^ signaling pathway. This causes the reversal of EMT, decreases chemoresistance, and eventually decreases self-renewal of the glioma stem cells to promote apoptosis.
(TIFF)
